# Microglia: An Interface between the Loss of Neuroplasticity and Depression

**DOI:** 10.3389/fncel.2017.00270

**Published:** 2017-09-08

**Authors:** Gaurav Singhal, Bernhard T. Baune

**Affiliations:** Psychiatric Neuroscience Lab, Discipline of Psychiatry, University of Adelaide Adelaide, SA, Australia

**Keywords:** glial cells, microglia, depression, cytokines, neuroprotection, neurodegeneration, immune

## Abstract

Depression has been widely accepted as a major psychiatric disease affecting nearly 350 million people worldwide. Research focus is now shifting from studying the extrinsic and social factors of depression to the underlying molecular causes. Microglial activity is shown to be associated with pathological conditions, such as psychological stress, pathological aging, and chronic infections. These are primary immune effector cells in the CNS and regulate the extensive dialogue between the nervous and the immune systems in response to different immunological, physiological, and psychological stressors. Studies have suggested that during stress and pathologies, microglia play a significant role in the disruption of neuroplasticity and have detrimental effects on neuroprotection causing neuroinflammation and exacerbation of depression. After a systematic search of literature databases, relevant articles on the microglial regulation of bidirectional neuroimmune pathways affecting neuroplasticity and leading to depression were reviewed. Although, several hypotheses have been proposed for the microglial role in the onset of depression, it is clear that all molecular pathways to depression are linked through microglia-associated neuroinflammation and hippocampal degeneration. Molecular factors such as an excess of glucocorticoids and changes in gene expression of neurotrophic factors, as well as neuro active substances secreted by gut microbiota have also been shown to affect microglial morphology and phenotype resulting in depression. This review aims to critically analyze the various molecular pathways associated with the microglial role in depression.

## Introduction

Depression is a common psychiatric disease prevalent worldwide and is associated with decreased life span and impaired quality of life (Bosnyák et al., 2015; Wachholz et al., 2016). One in every six people in the US is diagnosed with some form of depression sometime in his life (LB, 2014). A recent epidemiological study suggests that one is four women and one in six men suffer from depression at some stage of their life and depression is more prevalent in young people than elderly (Kessler et al., 2010). A door to door cross sectional study has confirmed that depression in elderly people resulted in increased morbidity and mortality, more significantly in females than males, in people who are single or divorced, lower in education, earning low income, unemployed, lacking health insurance, and suffering from other comorbid illnesses such as chronic obstructive pulmonary disease and cardiovascular diseases (Yaka et al., 2014). While depression is treatable, less that third of patients showed improvement in the immediate 18 months in secondary and tertiary care (Mulder et al., 2009).

The molecular mechanisms underlying the physiological symptoms of the disease have not been completely deciphered yet. Scientists around the globe have largely focused on serotonergic dysfunctions and cortisol dysregulation (Maes et al., 2009). However, due to the lack of sufficient evidence, the focus is now shifting onto the role of glial cells in the pathophysiology of depression. While neurobiological changes during depression, such as loss of neuroplasticity and neuroprotection, are being studied in detail (Fuchs et al., 2004; Pittenger and Duman, 2008; Player et al., 2013; Malykhin and Coupland, 2015), the involvement of glial cells in triggering changes in the brain remains to be fully understood.

Exploring the innate immune functions of glial cells is crucial to understand the role of brain's immune system to fight against the inflammatory and degenerative disorders. It further helps understand how does it protect the nerve cells, mediate neurobiological homeostasis, and further maintain the behavioral competency under normal conditions (Kreutzberg, 1995; do Carmo Cunha et al., 2007). Studies have shown that these cells are responsible for inflammatory and degenerative changes in the brain during aging (Schipper, 1996; Conde and Streit, 2006), psychological stress (Avitsur et al., 2005), ischemia (Nedergaard and Dirnagl, 2005; Shichita et al., 2012), and in the presence of harmful metabolites such as amyloid-β and tau peptides (Nagele et al., 2004). These cells also play a significant role in disruption of neuroplasticity and exacerbation of depression during psychological stress (Kreisel et al., 2014b).

Among glial cells, microglia have been shown to prominently express various cytokines which are essential for the maintenance of neurobiological homeostasis (Rothwell et al., 1996; Hanisch, 2002). Microglia exerts various opposing biological effects in the brain depending on their status and degree of activity in response to stimulus (Schwartz et al., 2006). They regulate activation and progression of various neuroimmune pathways that are mediated by immune components, such as natural killer cells, macrophages, T- and B-lymphocytes, cytokines, chemokines, Toll-like receptors, and growth factors. Activated microglia also initiate the formation of intracellular multiprotein complexes called as inflammasomes which in turn cleave precursor forms of IL-1β into its active form (Singhal et al., 2014). These immune cells and proteins in their physiological state are essential for the immune and tissue repair processes and the maintenance of neural-immune homeostasis during infectious diseases, trauma, ischemia, brain tumors, and autoimmune disorders. However, when over-expressed, they can cause a significant increase in the production and expression of proinflammatory cytokines (e.g., TNF-α, IL-1β) and neurotoxic substances (e.g., reactive oxygen species, nitric oxide), become increasingly dysfunctional and lose neuroprotective properties. Together, these may result in neuroinflammatory and neurodegenerative processes, subsequently leading to cognitive dysfunction and psychiatric illnesses, such as depression (Patel, 2013) and Alzheimer's disease (AD) (Mrak, 2012).

In addition to regulating immune functions, microglia have been reported to regulate various neurobiological processes, for example, formation of neural circuits (Wake et al., 2013) and synapses (Kettenmann et al., 2013) during early postnatal life, and phagocytose apoptotic cells in adult life (Sierra et al., 2010). Furthermore, microglia have been shown to regulate the levels of neurotrophic (Nakajima et al., 2007) and angiogenic factors (Rymo et al., 2011), and amino acids metabolism (Gras et al., 2012) in CNS. All these processes are vital for the sustenance of neuroplasticity and therefore may get compromised when microglia are reduced in number or become dysfunctional.

Other molecular factors, such as excess of glucocorticoids which have effects on microglial morphology and phenotype, have also been shown to result in depression (Nair and Bonneau, 2006; Marques et al., 2009). It has been shown that the density of neuroprotective microglia reduces in the dentate gyrus of the hippocampus (Branchi et al., 2014), prefrontal cortex (Hinwood et al., 2012), and amygdala (Hamidi et al., 2004) with chronic stress. In addition, microglia become increasingly dysfunctional and overexpress proinflammatory cytokines, class I and II major histocompatibility complex (MHC) antigens and toxic molecules (e.g., superoxide anions, nitric oxide) which lead to episodes of depression. Stress has also been shown to affect the composition of gut microbiota, which in turn could affect microglial activity leading to depression (O'Mahony et al., 2009; Erny et al., 2015).

Microglia, as immune regulatory cells in the brain, have received a great deal of attention in last two decades. However, their role in depression is yet to be fully elucidated and hence merits more research. This review, therefore, focuses on microglia and associated cytokines in the brain, their complex mechanisms of action, the intrinsic and extrinsic factors that trigger their activation and the key inflammatory pathways associated with microglia expression post-activation associated with depression.

## Materials and methods

### PRISMA criteria

Guidelines as prescribed by PRISMA (Preferred reporting items for systematic reviews and meta-analyses) were followed while constructing this review (Liberati et al., 2009; Moher et al., 2009). The checklist items from PRISMA as relevant to this review, for example those related to search and writing approaches, were included and the items not relevant, for example those related to meta-analyses, were excluded.

### Search and selection process

Electronic database search of PubMed, ScienceDirect and Google Scholar was systematically performed from January-1988 to March-2017 using various combinations of the following keywords: glial cells, microglia, depression, brain, CNS, astrocytes, neurogenesis, neurodegeneration, neuroprotection, neuroinflammation, neuroregeneration, cytokines, IL, TNF, TGF, chemokines, CRP, cellular, humoral, immune, aging, Alzheimer's disease, cognition, behavior, metabolic disorders, diabetes, obesity, cardiovascular disease, cancer, systemic, tryptophan, inflammasomes, NLRP3, hippocampus, cerebral, frontal cortex, pathogen-associated molecular patterns, and damage associated molecular patterns. At each stage of the search, titles and abstracts were scrutinized, and the most appropriate of them were organized into separate folders using EndNote X6.0.1 software (Clarivate Analytics). Articles relevant to our discussion were also retrieved from the reference list of other online articles on each subtopic. All duplicate articles in EndNote were then deleted. Articles without the full text available and with anecdotal evidence were excluded from the review.

The process mentioned above of Article selection and deletion yielded 1,784 articles in total. After placing all inclusion and exclusion criteria into our search (as depicted in Figure 1), a total of 412 full-text manuscripts were short-listed for further analysis. Both human and rodent data were included. In the next stages, 206 studies were further excluded following exclusion criteria as per Figure 1. In all, 206 articles closely related to the aims set forth for this review were selected and hence utilized.

**Figure 1:** Study inclusion flowchart. The flowchart depicts the systematic methodology for search and inclusion of relevant articles according to the PRISMA guidelines (Liberati et al., 2009; Moher et al., 2009).

### Inclusion and exclusion criteria

The various neuroimmune signaling pathways associated with microglial and microglia-derived cytokines activity in the brain and their association with depression have been critically analyzed in the current review. Hence the articles investigating immune functions of the microglia, their mechanism of actions during bidirectional communication between the nervous and immune systems and their association with depression were selected for detailed analysis.

## Depression as a psychiatric syndrome

Depression is characterized by psychophysiological changes, such as the state of low mood, losing the sense of self, sadness, irritability, and loss of interest in all activities and events (Belmaker and Agam, 2008). It is a major public health sector liability with an estimated economic burden of more than 80 billion dollars as was reported in 2000 (Donohue and Pincus, 2007). However, depression can be treated by optimal treatment.

Clinical depression or major depressive disorder (MDD) is the clinical manifestation of depressive state in humans and can be defined as the psychiatric syndrome characterized by the symptoms defined by the Diagnostic and Statistical Manual-5 (DSM-V) (see **Appendix I**; American Psychiatric Association, 2013). Most adults may have, at some point in their lives, experienced mood disorder in excess to physiologic changes and the majority of them may consult a primary care physician or a mental health professional. Depression alone has been the cause of wide scale mortality, in particular, due to suicides. According to a survey in the United States, MDD has led to higher suicidal rates in males than females (JL, 2015). Patients with MDD are more prone to develop life-threatening metabolic disorders such as type II diabetes and cardiovascular disease, further adding to mortality rates (Knol et al., 2006; Glassman, 2008). Indeed, unipolar depression is projected to be the second leading cause of disability worldwide in next two decades (González et al., 2010). However, it has been noted that 70–80% of individuals with MDD, if treated appropriately, recover to an appreciable extent (JL, 2015).

### Pathophysiology of depression

Clinical depression seems to occur more commonly in people with certain risk factors (Kendler et al., 2006a). Besides external and environmental factors like substance abuse, lack of peer support, marital problems, low socioeconomic status, low education, and stressful life events; many of the internalizing factors play a major role as well. Significant among them are genetic alterations and acquired anatomical defects. Certain genetic subgroups are more vulnerable to developing depression, and monozygotic twins show a concordance rate of almost 40% for developing MDD (Sullivan et al., 2000; Kendler et al., 2006b). In spite of observed anatomic and physiologic changes in brain, no conclusive proof has been found linking any combination of genetic and environmental factors (aan het Rot et al., 2009; Risch et al., 2009). The altered levels in certain growth factors and neurotransmitters such as serotonin, norepinephrine, dopamine, GABA, brain-derived neurotrophic factor (BDNF), glutamate, cannabinoid (CB1) receptors, acetylcholine, and substance P have been proven time and again to cause depression and the protocols for treating depression have been developed to maintain those imbalances (Duman et al., 1997; Svenningsson et al., 2006; Thase, 2007; Hill and Gorzalka, 2009). Also, factors like over and under activity of hypothalamic-pituitary-adrenal axis may also be responsible for MDD (Gillespie and Nemeroff, 2005; Vreeburg et al., 2009). However, researchers have found that these functional causes go hand-in-hand with anatomic alterations at the cellular level (Rajkowska and Miguel-Hidalgo, 2007).

### Role of cellular alterations in pathogenesis of depression

Several anatomical changes are related to depression as detected in magnetic resonance studies of the brain (Koolschijn et al., 2009). Some of the consistent findings are decreased lobar volumes, especially frontal, temporal, and hippocampal volumes and higher volumes of ventricles on overall brain volume (Lampe et al., 2003; Taylor et al., 2007). There is a significant loss of GABAergic neurons in occipital, prefrontal and limbic regions and size of neurons are decreased by one-fifth (Cotter et al., 2001, 2002; Rajkowska et al., 2007; MacIag et al., 2010). Significant changes are noted in the number, density and size of glial cells during MDD (Ye et al., 2011). These evidences suggest the role of glial cells in mood disorders and the potential part played in the pathogenesis of the latter. We, however, limit our discussion to microglia among the glial cell population and their effects post activation leading to depression in this review.

## Microglia: multitasking cells of the brain

Microglia comprises of about 7–10% of all brain cells, and are involved in maintaining the development and normal structural and functional processes of neurons. They are non-excitable cells of mesodermal origin, and together with other glial cells, such as astrocytes and oligodendrocytes, they form the smaller but numerous (in comparison to neurons) clusters of cells in the CNS (Brown et al., 1997; Zhang, 2001). Microglia assist with neuronal migration during brain development, repair damaged neurons, fill voids left by degenerative neurons, recycle neurotransmitters after neuronal excitation, regulate ionic balance, buffer pH, phagocytize dead cells and pathogens, and express various immune proteins and cell adhesion molecules required for the initiation of the innate immune response in the presence of pathogens and stress proteins (Bunge, 1994; Zhang, 2001; Kitamura and Nomura, 2003).

## Modulation of neuroimmune response by microglia

Microglia are the principal immune effector of the brain responsible for immunosurveillance and neuroprotection. Microglia, in association with cytotoxic T cells, are important for neurogenesis, adult brain plasticity and spatial memory (Ziv et al., 2006). While sessile in the CNS, the quiescent forms of microglia lack phenotypical markers required for antigen presentation, suggesting that their activation is tightly regulated to prevent any autoimmune reactions under normal conditions. Once activated in the presence of pathogens associated molecular patterns (PAMPs) and/or damage associated molecular patterns (DAMPs), they rapidly proliferate and express MHC class I and MHC class II proteins, receptors for various proinflammatory cytokines, toll-like receptors, Nod-like receptors, and antigens for T-cells subsets essential to mount innate immune response (Dodel et al., 2004). The microglial activity is further triggered by the infiltrating hematogenous macrophages which find a way to the CNS when the endothelial cells lining of the blood brain barrier is ruptured during brain injuries and pathologies (Dong et al., 2002).

The overexpression of proinflammatory cytokines in the brain and influx of immune phagocytic cells is essential to control brain damage and promote faster healing, however it has also been shown to contribute toward neurodegeneration and hence playing an important role in the pathophysiology of brain diseases such as depression, dementia and AD in clinical trials (Cacquevel et al., 2004; McAfoose and Baune, 2009; You et al., 2011). However, when the stimulus diminishes, microglia produce, and express anti-inflammatory cytokines causing microglial apoptosis and disintegration of proinflammatory cytokines, thereby switching off the immune response to stimulus (Garden and Möller, 2006).

Microglia numbers increase in the brain of aging rodents and are, subsequently, found to be related to cognitive and memory impairment (Sugaya et al., 1996; Rozovsky et al., 1998), neuropsychiatric disorders such as depression (Norden and Godbout, 2013) and neurodegenerative diseases such as AD (Mrak and Griffin, 2005). They become increasingly dysfunctional and loses their neuroprotective properties with age, and release excessive quantities of proinflammatory cytokines when stimulated by PAMPs and DAMPs. In association with genetic factors and acquired environmental risks, this predisposes the brain to the development of aging-associated psychiatric disorders (Mrak and Griffin, 2005; Streit, 2005; Dilger and Johnson, 2008; Norden and Godbout, 2013). Interestingly, this phenomenon during aging has been observed to occur more prominently in the hippocampus than in the cerebral cortex affecting both cognition and memory (Xie et al., 2003).

## Role of microglia expressed cytokines in the CNS

Microglia, along with astrocytes, prominently express various proinflammatory and anti-inflammatory cytokines in the brain and hence any action of these cytokines can primarily be associated with microglial activity in the CNS.

Proinflammatory cytokines, such as TNF-α and IL-1β attract leucocytes and enhance their proliferation. They also stimulate cytotoxicity, the release of proteolytic enzymes, synthesis of prostaglandins and initiate synthesis and secretion of secondary cytokines which in turn promote inflammation and increases thermoregulatory set point (Cannon, 2000). Also, certain chemokines (e.g., IL-8) facilitate passage of leucocytes from circulation into the surrounding tissues and enhance inflammation (Kushi et al., 2003). Similarly, the monocyte chemotactic protein (MCP) family including CCL2, CCL7, CCL8, CCL12, and CCL13 (designated MCP 1–5, respectively) exert potent proinflammatory actions through chemotaxis of monocyte-derived macrophages and other inflammatory leukocytes to the inflamed or injured CNS (Yamagami et al., 1999). Also, IL-1 and TNF-α secrete adhesion molecules that attach to the endothelium of blood vessels in the brain and facilitate migration of leucocytes from blood to the brain tissues (Kim, 1996).

In contrast, research has shown that anti-inflammatory cytokines modulate the expression of genes responsible for proinflammatory cytokines production, in turn regulating inflammatory response. For example, transgenic mice deficient in or knocked out for genes transcribing anti-inflammatory cytokines, such as IL-1ra, IL-10, and TGF-β1 showed enhanced inflammatory reactions (Dinarello, 2000). Interestingly, TGF-β KO mice were found to be devoid of microglia suggesting that TGF-β is important for the formation of microglia and neuroimmune regulation during brain diseases (Butovsky et al., 2014).

Levels of both proinflammatory and anti-inflammatory cytokines have been shown to elevate in depression, resulting in cognitive and memory deficit (Kronfol and Remick, 2014). However, cytokines alone may not be responsible for these adverse changes, and a combination of various chemokines and cytokines may be the cause (Baune et al., 2009).

## Elevated peripheral proinflammatory cytokines level → movement to brain

Prospective and correlation studies have established an association between the high incidences of chronic inflammatory diseases such as cancer (Il'yasova et al., 2005), diabetes (De Rekeneire et al., 2006), osteoarthritis (Stannus et al., 2013), and cardiovascular disease (Volpato et al., 2001) in aged cohort with increased levels of systemic proinflammatory cytokines such as TNF-α, IL-1β, and IL-6 and acute phase proteins (e.g., C-reactive protein; CRP). Also, there is a significant association between age-related depression and the levels of proinflammatory cytokines in the brain (Godbout et al., 2008). This suggests that some pathways may be responsible for the movement of proinflammatory cytokines from the systemic circulation to brain parenchyma leading to depression during metabolic chronic inflammatory disorders. Three such pathways viz. humoral, neural, and cellular pathways have been proposed by Capuron and Miller (2011). The specific role of these pathways in the comorbidity of chronic inflammatory systemic diseases with psychiatric disorders is not yet fully elucidated and hence calls for more research.

## Role of blood-brain-barrier in cross immune-regulation and microglial activation

Studies on rodents show that activated T cells migrate across the blood-brain-barrier (BBB) during neuroinflammation and are present at all times in the brain along with macrophages/monocytes for immune surveillance (Hickey et al., 1991; Engelhardt, 2006). It is contrary to the long-standing view that BBB provides an immune privileged status to the brain. The CD4+ T helper (Th) 1 cells secrete proinflammatory cytokines in the brain on stimulation with pathogens and stress proteins which, in turn, activate macrophages and microglia-driven cell-mediated immune response resulting in inflammatory condition (Fiorentino et al., 1989; Dinarello, 2000). CD4+ Th2 cells thereafter produce anti-inflammatory cytokines, which activate humoral immune system (activate B lymphocytes) suppressing microglia and subsequent production of proinflammatory cytokines IL-1β and TNF-α, and chemokines such as IL-8 and vascular adhesion molecules, thereby reducing neuroinflammation (Fiorentino et al., 1989; Dinarello, 2000).

## Critical analysis of the hypotheses elucidating role of microglia in depression

Various molecular hypotheses elucidating the role of microglia in depression are interconnected and essentially go through neuroinflammation and hippocampal degeneration before they lead to the development of depression (see Figure 2). These are discussed and critically analyzed below.

**Figure 2:** Different hypotheses for depression converge together and are interconnected. As seen in the figure, microglia can cause depression through different molecular pathways. These mechanistic pathways are sometimes interrelated making the whole mechanistic link between microglial action and depression complex. Red boxes indicate “neuroinflammatory pathway,” gray boxes indicate “altered neurotrophin levels pathway,” and “impaired hippocampal neurogenesis pathway,” blue boxes indicate “altered brain tryptophan metabolism pathway,” green boxes indicate “stimulation of peripheral immune system pathway,” brown boxes indicate “psychological/chronic stress and reduced immunity pathway,” and purple boxes indicate “Inflammasome pathway.” Black boxes are part of more than one pathways. IFN, interferon; TNF, tumor necrosis factor; IL, interleukin; P2X7, two-transmembrane ATP-gated ionotropic purinoreceptor; CVD, cardiovascular disease; LPS, lipopolysaccharide; PAMPs, pathogen-associated molecular patterns; DAMPs, damage-associated molecular patterns; CNS, central nervous system; TBI, traumatic brain injury; IDO, indoleamine 2, 3-dioxygenase enzyme; KP, kynurenine pathway.

### The neuroinflammatory hypothesis

Microglia overexpress proinflammatory cytokines in the CNS in response to adverse stimuli, such as psychological stress (Avitsur et al., 2005; You et al., 2011), age (Kumagai et al., 2007), metabolic disorders (Volpato et al., 2001; Il'yasova et al., 2005; De Rekeneire et al., 2006; Stannus et al., 2013), traumatic brain injuries (Fenn et al., 2014), or infections (Dunn, 2006). This results in neuroinflammation, leading to an imbalance of several brain functions, some of them being the characteristics of MDD as per DSM-V, such as low mood, insomnia, fatigue and change in appetite (Maes et al., 1997; Howren et al., 2009; Dowlati et al., 2010; Hannestad et al., 2011). A recently conducted study has shown that microglia get primed with MHC II complex and overexpress proinflammatory cytokines even post 30 days after traumatic brain injury in BALB/c mice. These changes in microglial morphology has been found to be associated with depressive-like behavior (Fenn et al., 2014). A meta-analysis reported high concentrations of the proinflammatory cytokines TNF-α and IL-1β and IL-6 in depressed subjects than controlled subjects (Dowlati et al., 2010). These findings are consistent with the previously published reviews and may be associated with the hyperactivity of microglia in the brain (Hanisch, 2002; Schroeter et al., 2008; Smith et al., 2012). TNF-α produced in response to microglial hyperactivity causes hippocampal degeneration and microglial apoptosis (Cacci et al., 2005), the former being a characteristic finding in patients with unipolar depression (Videbech and Ravnkilde, 2015). In addition, IFN-α promotes expression of proinflammatory surface markers MHC II, CD86, and CD54 indicating M1 polarization, thus leading to neuroinflammation and depression (Wachholz et al., 2016). All above pathways associate alterations in microglial morphology and activity to neuroinflammation which subsequently lead to the development of depression.

Contrary to above, when the inflammatory response is blocked with external non-steroidal anti-inflammatory factors, such as Indomethacin and Ibuprofen, and with fusion proteins produced from recombinant DNA, such as Etanercept that inhibits microglial TNF expression (lou Camara et al., 2015), a considerable improvement in neurogenesis (Monje et al., 2003) and a reduction in depressive-like behavior (Iyengar et al., 2013) has been reported. Antidepressants such as imipramine and minocycline reduce proinflammatory cytokines levels by inhibiting microglial proliferation and activation, and subsequently attenuate depressive-like symptoms (Tikka et al., 2001; Fischer et al., 2015; Zheng et al., 2015). Imipramine has been shown to reduce the number of chronic stress induced- activated hippocampal microglia (Iwata et al., 2016), perhaps by selectively inhibiting the M1 polarization of microglia (Kobayashi et al., 2013). Similarly, another antidepressant, pioglitazone acts by inhibiting the increased numbers and microglial morphological alterations in the hippocampus, reducing the overexpressing microglial M1 markers and increasing the under-expressed microglial M2 markers in C57BL/6 mice exposed to chronic mild stress (Zhao et al., 2016). Another technique involves using transgenic proinflammatory cytokines receptor antagonists, such as IL-1 receptor antagonist that reduces microglial apoptosis and subsequently neuroinflammation and depressive-like behavior in rodents (Goshen et al., 2008; Koo and Duman, 2009; Kreisel et al., 2014a). Neuroinflammation, therefore, is one of the main etiological factor for depression and most currently available treatments for depression alter the related pathways, in turn, alleviating inflammation in brain.

### Inflammasome hypothesis

The inflammasomes hypotheses of depression and its comorbidity with systemic illnesses have been reviewed elsewhere (Iwata et al., 2013; Singhal et al., 2014). Inflammasomes are cytosolic protein complexes which when assembled and activated in the presence of PAMPs and DAMPs, further activate proinflammatory caspases, in particular, caspase-1. Caspase 1 subsequently splits inactive forms of proinflammatory cytokines IL-1β, IL-18, and IL-33 into their active forms (Arend et al., 2008; Chakraborty et al., 2010) causing neuroinflammation (Davis et al., 2011) which is the leading etiology of depression as mentioned previously (Walker et al., 2014). The role of microglia is important in the activation of inflammasomes as they carry pattern recognition receptors (PRRs) that function to recognize PAMPs and DAMPs. While PRRs can be membrane bound (toll-like receptors) or localized within the cytoplasm Nod-like receptors (NLRs), it is the NLRs which when activated lead to the assembly and activation of inflammasomes in the cytoplasm (Arend et al., 2008; Chakraborty et al., 2010). Of all inflammasomes, NLRP (Nod-like receptor family, containing pyrin domain) inflammasomes have been primarily implicated in the etiology of depression (Zhang Y. et al., 2014; Ghisleni, 2017; Kaufmann et al., 2017). The microglial membrane is rich in purinergic receptor P2X7 which when activated with chronic stress subsequently activates NLRP3 inflammasome in hippocampal microglia augmenting proinflammatory environment in the CNS (Yue et al., 2017). A study has confirmed the role of NLRP3 inflammasomes in lipopolysaccharide (LPS)-induced depressive-like behavior in mice (Zhang Y. et al., 2014). Similar findings were seen in human participants when activated NLRP3 inflammasomes were detected in blood mononuclear cells from depressive patients (Alcocer-Gómez et al., 2013). Interestingly, TNF-α has also been shown to trigger the activation of caspase 1 and in turn secretion of IL-1β from microglia (Alvarez and Munoz-Fernandez, 2013), further aggravating neuroinflammation. Interestingly, it has been suggested that inflammasome-related inflammation is an ongoing process in psychiatric patients during disease states (Hohmann et al., 2014).

The finding that mice lacking caspase-1 are resistant to LPS-induced depressive-like behavior further supports the above inflammasome hypotheses for depression (Moon et al., 2009). Based on this, targeted therapies such as antidepressants like fluoxetine which alleviate depression by inhibiting the peripheral and central NLRP3 inflammasome activation have been developed (Du et al., 2016). Chrysophanol also exerts similar effects, however by inhibiting P2X7 pathway (Zhang et al., 2016), and hence plausibly the subsequent activation of NLRP3 inflammasome as mentioned earlier.

### Stimulation of peripheral immune system hypothesis

Increased levels of systemic proinflammatory cytokines and acute phase proteins (e.g., C-reactive protein) have been reported in chronic inflammatory diseases such as cancer (Il'yasova et al., 2005), diabetes (De Rekeneire et al., 2006), osteoarthritis (Stannus et al., 2013), and cardiovascular disease (Volpato et al., 2001) in aged cohorts. An association between age-related depression and level of proinflammatory cytokines in the brain has also been established (Godbout et al., 2008). These findings hint to a possible mechanism whereby proinflammatory cytokines and acute phase proteins play a crucial role in the comorbidity of systemic diseases with depression, especially during old age. To support this hypothesis, a look back is required into a previously published review describing various pathways for the transport of proinflammatory cytokines to brain from systemic circulation (Capuron and Miller, 2011). In one of the pathways, cellular pathway, TNF-α secreted from activated monocytes and macrophages migrates to brain through BBB and stimulates microglia to produce MCP-1, in turn recruiting monocytes into the brain. Also, increased production and expression of IL-1β in the brain after LPS-induced systemic inflammation (Cunningham et al., 2005) and changes in mood and behavior similar to depression after systemic administration of proinflammatory cytokines (Pollak and Yirmiya, 2002) has been reported in rodents. Given that metabolic disorders can predispose to the development of psychiatric disorders, it is possible that inflammasome-driven inflammatory pathways in the cytoplasm of microglia may be a potential mechanism driving this co-morbidity as these pathways have been shown to be associated with the development of Type II diabetes (Grant and Dixit, 2013; Lee et al., 2013), obesity (Stienstra et al., 2011), and cardiovascular diseases (Garg, 2011), as well as cancer (Zitvogel et al., 2012). The activation of inflammasomes in microglia, particularly NLRP3, therefore could be indirectly related to the pathophysiology of depression and its comorbidity with other systemic diseases through an inflammatory response in the brain.

### Psychological stress and reduced immunity hypothesis

Recent studies have established a causal relationship between the stress-related life events/chronic stress and depressive-like behavior in mice (Goshen et al., 2008; Berry et al., 2012). Indeed, chronic unpredictable mild stress (CUMS) has been shown to cause neuroinflammation and subsequently depression in several studies (Farooq et al., 2012; Ramirez et al., 2016; Tong et al., 2017). Microglial dysfunction has been implicated in chronic unpredictable stress-induced neuroinflammation and depression-like condition in rodents (Kreisel et al., 2014a). In a study, the initial phase of stress stimulation induced microglial proliferation and activation while prolonged stress resulted in microglial apoptosis leading to a reduction in their numbers, reduced expression of activation markers and dystrophic morphology in the hippocampus (Kreisel et al., 2014a). Microglia have been shown to get hyper-ramified during chronic stress leading to depression (Hellwig et al., 2016). It is interesting to note that microglial increase in numbers and transition from a ramified-resting state to a non-resting hyper-ramified state is more in certain stress-sensitive brain regions in response to the chronic stress (Tynan et al., 2010). Indeed, repeated chronic stress increased numbers of hyper-ramified microglia in the hippocampus, prefrontal cortex, amygdala, and nucleus accumbens (Bian et al., 2012; Farooq et al., 2012; Wohleb et al., 2012; Kopp et al., 2013). Hyperactivated microglia produce excessive proinflammatory cytokines, show enhanced antigen presentation and become increasingly phagocytic (De Pablos et al., 2006; Bradesi et al., 2009; Giovanoli et al., 2013; Lehmann et al., 2016). In addition, microglial response to stress proteins is guided by their glucocorticoids receptors (Frank et al., 2012) and nor-adrenaline activated alpha/beta-adrenergic receptor signaling pathways (Blandino et al., 2006). For example, stress hormones down-regulate glucocorticoids receptors which further declines microglial response to the stress proteins (Reichardt et al., 2001; Cohen et al., 2012). Similarly, a decline in the secretions of proinflammatory cytokines from microglia has been reported in response to nor adrenaline-activated alpha/beta-adrenergic receptor signaling pathways (Mori et al., 2002; Russo et al., 2004; Färber et al., 2005; O'Sullivan et al., 2009).

Evidently, few antidepressants have been shown to exert anti-depressive effects by restoring microglial morphology to the resting stage. For example, chronic treatment with the antidepressant venlafaxine restored microglia morphology and reduced depression-like behavior (Hellwig et al., 2016). Likewise, blocking of initial proliferation and activation of microglia in response to CUMS using antidepressants minocycline and imipramine prevented subsequent apoptosis and morphological distortions of microglia and hence depressive behavior (Kreisel et al., 2014a).

### Alteration in brain tryptophan metabolism hypothesis

Many recent studies have found a link between MDD and activation of the enzymes indoleamine 2, 3-dioxygenase (IDO), and signaling via the kynurenine pathway (KP) (Dantzer, 2016; Parrott et al., 2016; Liu et al., 2017). Microglial IDO is activated by inflammatory cytokines like IL-6, TNFα, IFN-γ, and their inducers like LPS and HIV Tat protein (Dantzer et al., 2011; Walker et al., 2013). The involvement of the microglial KP in mediating inflammation and stress-induced depression is supported by clinical studies demonstrating that IFN-α immunotherapy increases tryptophan metabolism through the KP pathway, both in periphery and CSF, and this increase is significantly correlated with the development and severity of IFN-α-induced depression (Capuron et al., 2003). A recent clinical trial investigated cerebral tryptophan metabolism in brain-tumor associated depression and established that abnormalities in tryptophan transport and metabolism in the thalamus, striatum, and frontal cortex are associated with depression in patients which may, in turn, indicate an imbalance between the serotonin and kynurenine pathways (Bosnyák et al., 2015). Although, research in this direction is still in infancy stage, altering tryptophan metabolism pathways has shown good potential in treating depression in recent times (Abildgaard et al., 2017; Eskelund et al., 2017).

### Altered neurotrophins (BDNF and GDNF) levels hypothesis

Microglia are known to modulate the production of neurotrophins, mainly BDNF (Ferrini and De Koninck, 2013), a protein known for regulating neurogenesis in the dentate gyrus of the hippocampus (Rossi et al., 2006; Fan et al., 2007) and enhancing dendritic branching (McAllister et al., 1995; Horch and Katz, 2002; Horch, 2004). It is widely known to be associated with hippocampal plasticity (Ye et al., 2011). Neurotrophin deficiency in the presence of dystrophic microglia may therefore hinder hippocampal neurogenesis and further precipitate depressive-like symptoms.

BDNF infusion is seen to partially reverse the effect of the chronic stress-induced depressive behavior in a rat model (Ye et al., 2011). The use of Gastrodin and total glycosides of peony (TGP), both of which are Chinese herbs used to treat depression, as well as the antidepressants like imipramine and fluoxetine are seen to up-regulate the hippocampal BDNF mRNA expression (Mao et al., 2010; Takano et al., 2012; Quesseveur et al., 2013; Zhang R. et al., 2014). On the other hand, an overexpression of BDNF also has an anxiolytic effect and promotes local neurogenesis (Quesseveur et al., 2013). Similar effects of these drugs are seen on the up-regulation of Glial Cell Line-derived Neurotrophic Factor (GDNF) (Hisaoka-Nakashima et al., 2015). The role of GDNF in depression was further supported by lower serum GDNF concentrations in MDD patients as compared to controls (Zhang et al., 2008).

### Impaired hippocampal neurogenesis hypothesis

The role of microglia in hippocampal neurogenesis has been discussed many times in the past, and hence we have limited our discussion to few important points on this topic for the purpose of this review. Impaired hippocampal neurogenesis has been shown to be an important underlying cause of depression (Jacobs et al., 2000). Numerous studies have reported that microglia activation plays a key role in suppression of hippocampal neurogenesis under conditions of stress and inflammation (Kempermann and Neumann, 2003; Sierra et al., 2014). Studies on mice have shown that irradiation or treatment with lipopolysaccharide causes marked suppression of hippocampal neurogenesis, while treatment with minocycline negated this effect (Ekdahl et al., 2003; Monje et al., 2003). Interestingly, neurogenesis suppression in response to microglial activation was primarily due to the detrimental effect on maintenance of newborn neurons rather than on their proliferation (Ekdahl et al., 2003; Monje et al., 2003). Further, *in-vitro* experiments have shown that the conditioned media from LPS-challenged microglia induced IL-6 or TNFα-mediated apoptosis in hippocampal neuroblasts (Monje et al., 2003; Cacci et al., 2005). These findings therefore suggest that hippocampal neurogenesis is affected by the microglial activation status. Although, hippocampal degeneration has been shown to result primarily in response to chronic neuroinflammation during aging, the exact mechanism for the same is still not elucidated.

### Recent evidence to support the role of microglia in depression

Recent evidence has confirmed that both over expressed and under expressed microglia can cause depression. While over expressed microglia trigger the onset of depression through the neuroinflammatory pathway as mentioned before, under expressed microglia could result in depression through hippocampal degeneration pathway. Chronic form of stressors, for example chronic unpredictable stress, chronic restraint stress, and chronic social defeat stress have all lead to depression through reduction in the number of hippocampal microglia (Tong et al., 2017). On the other hand, rats exposed to learned helplessness showed increase in the number of activated microglia in the granule cell layer, hilus, CA1, and CA3 regions of the hippocampus (Iwata et al., 2016). Overall, this suggests that both the under expression and over expression of microglia in brain lead to depression albeit through different molecular pathways. As such, altering these molecular pathways associated with microglial activity through pharmacological and non-pharmacological means could provide a novel therapeutic intervention for depression.

Indeed, some recent studies have shown that treatment with antidepressants Imipramine or Minocycline decreases IFN-γ levels by inhibiting microglial activation and subsequently reduces the depressive symptoms in animal models of depression (Fischer et al., 2015; Zheng et al., 2015). Studies involving a transgenic IL-1 receptor antagonist have shown to reduce microglial apoptosis and subsequently neuroinflammation and depressive-like behavior in rodents (Goshen et al., 2008; Koo and Duman, 2009; Kreisel et al., 2014a). Similarly, Etanercept, known to reduce depression associated with rheumatoid arthritis and psoriasis (Tyring et al., 2006; Kekow et al., 2009), has been shown to inhibit microglial TNF expression and reduce brain inflammation in C57BL/6 mice (lou Camara et al., 2015). These results clearly demonstrate the recent developments in microglia targeted therapies for depression.

More recently, the role of gut microbiota on the brain development, immunomodulation and change in behavior has attracted attention of researchers. While gut lining is impermeable to toxic substances, any microdamage to it could increase the permeability and movement of micro molecules both ways (Turner, 2009). Microorganisms, such as firmicutes, bacteroidetes, actinobacteria, and proteobacteria, that live in the intestine (Ley et al., 2006) interact with immune cells through the permeable mucosal lining forming bidirectional communication between the brain and the gut (Mayer, 2011). TLRs on the gut lining play a vital role in the initiation of this communication and passing the immune message to the brain (Zeuthen et al., 2008). Recent evidence has established the role of gut microbiota in the development of depression, perhaps through the production of neuroactive substances such as serotonin, nor-epinephrine, dopamine, and gamma-aminobutyric acid, which act on the gut-brain axis (Dinan and Cryan, 2013). Interestingly, current antibiotics treatment for infections, as well as vaccinations have been shown to affect the integrity of gut microbiome (Evrensel and Ceylan, 2015). If this has any effect on the development of depression is however still not established. In addition, stress can also influence the diversity of gut microbiota, for example decrease in the levels of fecal Lactobacillus was observed in rats separated from their mother (O'Mahony et al., 2009).

As we discussed above, change in microglial morphology and activity is hugely responsible for the onset of depression. Until recently, it was however not known if gut microbiota has any effect on microglia and associated development of depression. However, a research from Erny et al. has provided evidence for the role of gut microbiota in depression through modulation of microglial associated immune network. Researchers observed that germ free mice showed defects in microglial functions as well as reduction in their numbers, leading to impaired immune response affecting neural circuitry, a potential factor for the onset of depression (Erny et al., 2015). This overall suggest that gut microbiota has a role in the onset of depression, especially during early age, through the alteration of microglial activity in brain. However, further research is required to establish this hypothesis.

## Discussion

While psychiatry deals with patterns in behavior and cognition, neuroimmunology aims to understand the complex molecular biology of the brain behind those patterns. Much research has been conducted to uncover the physiological mechanisms behind depression using both animal and human models. However, due to the complex pathological and physiological nature of molecular events occurring during depression, difficulties arise when it comes to treatment and management strategies (see Figure 3). The role of microglia has been studied extensively over last decade, which has given the opportunity to our scientific community to devise ways of modulating their functions, preventing the development of depression and hence keeping the brain healthy. However, various functions of microglia have no precise boundaries and pose a multitude of questions till date.

**Figure 3:** Mechanistic pathways of some of the pharmacological interventions available currently to treat depression. The figure depicts mechanistic pathways of some of the pharmacological drugs that are shown to reduce the depressive-like behavior. IFN, interferon; P2X7, two-transmembrane ATP-gated ionotropic purinoreceptor. Different colors depict different mechanistic pathways of the drugs in reducing the depressive-like behavior. For example, red boxes indicate reduced M1 microglial polarization, microglial apoptosis, and morphological changes, brown boxes indicate enhanced hippocampal neurogenesis, gray boxes indicate restoration of microglial morphology to resting state, blue boxes indicate reduced neuroinflammation and neurodegeneration and green boxes indicate reduced inflammasome activation.

Microglia act as resident macrophages in the CNS and remain quiescent for most time that is required to save them from apoptosis and regular replacement (Gehrmann, 1996). However, their activation in the presence of infectious foreign matter, such as bacteria and viruses or metabolic by-products, such as Aβ, rapidly mount the necessary immune reaction (Nagele et al., 2004; Conde and Streit, 2006). Indeed, the biomarker to detect microglial functions, IBA-1 is the most reliable source to diagnose neurodegenerative conditions (Ahmed et al., 2007). Analysis of IBA1 marker when associated with a specific set of inter-correlating symptoms, distinguishable from other symptom groupings in other psychiatric disorders and sufficiently stable to allow predictions, can help to predict the course and treatment outcome for depression.

Overexpression of proinflammatory cytokines in microglia is one of the primary factors responsible for the development of depression in diverse situations (Volpato et al., 2001; Avitsur et al., 2005; Il'yasova et al., 2005; De Rekeneire et al., 2006; Dunn, 2006; Kumagai et al., 2007; You et al., 2011; Stannus et al., 2013; Fenn et al., 2014). The related underlying factors include inflammation of neurons (Kumagai et al., 2007), neurodegeneration and apoptosis (Cacci et al., 2005; Kumagai et al., 2007), impaired neurogenesis (Kempermann and Neumann, 2003; Sierra et al., 2014), production of stress proteins (Goshen et al., 2008; Berry et al., 2012; Ramirez et al., 2016; Tong et al., 2017), alteration in brain tryptophan (Bosnyák et al., 2015; Dantzer, 2016; Parrott et al., 2016; Liu et al., 2017), and neurotrophins metabolisms (Zhang et al., 2008; Ye et al., 2011; Ferrini and De Koninck, 2013), as well as morphological and functional changes in microglia itself (Fenn et al., 2014), all leading to depression. Also, instead of acting directly, microglia may first activate the inflammasomes in more glial cells, in turn releasing an IL-1 family of cytokines, causing neuroinflammation and depression (Arend et al., 2008; Chakraborty et al., 2010; Alcocer-Gómez et al., 2013; Zhang Y. et al., 2014), and this could be an ongoing process in psychiatric patients (Hohmann et al., 2014).

More significantly, microglia overexpressing proinflammatory cytokines could be responsible for the comorbidity of systemic metabolic diseases with depression (Volpato et al., 2001; Il'yasova et al., 2005; De Rekeneire et al., 2006; Godbout et al., 2008; Stannus et al., 2013). Moreover, it is now confirmed that T cells and proinflammatory cytokines can cross BBB (Hickey et al., 1991; Engelhardt, 2006) and microglia are associated with one of the pathways responsible for this transfer of proinflammatory cytokines from the systemic circulation to the CNS through BBB (Capuron and Miller, 2011). NLRP3 inflammasomes could play a major role in the comorbidity of depression with other systemic diseases, indirectly through an inflammatory response in the brain (Pollak and Yirmiya, 2002; Garg, 2011; Stienstra et al., 2011; Zitvogel et al., 2012; Grant and Dixit, 2013; Lee et al., 2013; Ghisleni, 2017; Kaufmann et al., 2017; Yue et al., 2017).

Our discussion above as well as some other reviews (Liu and Hong, 2003; Glezer et al., 2007; Ekdahl et al., 2009) suggest that microglia can display both neuroprotective and neurotoxic effects depending on the extent of their cytokines expression. However, this is also dependent on factors like aging, the presence of pathogens and stress proteins, and external environmental conditions. Different pharmacological interventions currently available for depression although block specific mechanistic pathways (see Figure 3), microglia can still be a potential target for further extensive research to develop a treatment providing fast and complete cure from depressive-like behavior with no or little side effects.

## Concluding remarks

The above discussion suggests that both immune and non-immune aspects of microglia impact on neurogenesis and neuroplasticity with either neuroprotective or detrimental effects depending on the condition. When detrimental, development of depressive-like behavior is a common phenomenon. Microglia, therefore, could be a potential target for the treatment of depression. Microglia-targeted therapeutic intervention in depression requires a complete understanding of molecular pathways leading to the activation and suppression of these glial cells and subsequent effects on neuroplasticity. Indeed, molecular pathways leading to the activation and suppression of microglia, and associated effects on immune cells and proteins, neuronal signaling, neural activation, neuronal plasticity, and behavioral endpoints have largely been unexplored yet and therefore calls for further extensive research.

## Author contributions

GS: Writing. BB: Writing, Proofreading, Supervising.

### Conflict of interest statement

The authors declare that the research was conducted in the absence of any commercial or financial relationships that could be construed as a potential conflict of interest.

## Appendix I

Diagnostic criteria for MDD as per DSM-V (American Psychiatric Association, 2013).

**Table:**

**Factor**	**Criteria**	**Time frame (if applicable)**
Mood	Loss of interest or pleasure in day to day activities	>2 weeks
Impaired function	Social, occupational, educational	–
**AT LEAST 5 OF THE FOLLOWING NINE MUST BE POSITIVE FOR MDD:**		
Depressed mood/irritable	Feeling sad/empty/tearful	Most of the day, nearly every day
Decreased interest/pleasure	Loss of interest in most daily activities	Most of each day
Significant weight change/Change in appetite	5% loss of weight	–
Change in sleep pattern	Insomnia/hypersomnia	–
Change in activity	Psychomotor agitation/retardation	–
Fatigue/Loss of energy	Feeling tired	Most of the time
Guilt/Worthlessness	Feeling of inappropriate guilt/worthlessness	–
Concentration	Unable to concentrate/indecisiveness	–
Suicidality	Thoughts/Plan of committing suicide	–
**OTHER SYMPTOMS OF DEPRESSION**		
Not able to relax, feeling tense all the time, unpleasant thoughts, fear of something awful that might happen.		
